# Antitumor Activity of lncRNA NBAT-1 via Inhibition of miR-4504 to Target to WWC3 in Oxaliplatin-Resistant Colorectal Carcinoma

**DOI:** 10.1155/2022/9121554

**Published:** 2022-04-21

**Authors:** Chen Li, Xu Li

**Affiliations:** ^1^Center for Translational Medicine, The First Affiliated Hospital of Xi'an Jiaotong University, Xi'an 710061, China; ^2^Molecular Testing Center, The First Affiliated Hospital of Jinzhou Medical University, Jinzhou 121001, China; ^3^Key Laboratory for Tumor Precision Medicine of Shaanxi Province, The First Affiliated Hospital of Xi'an Jiaotong University, Xi'an 710061, China; ^4^Key Laboratory of Environment and Genes Related to Diseases (Xi'an Jiaotong University), Ministry of Education of China, Xi'an 710048, China

## Abstract

**Background:**

Increasing evidence shows that dysfunction of noncoding RNAs is implicated in cancer. Neuroblastoma associated transcript 1 (NBAT-1) has been identified as a tumor suppressive lncRNA that is aberrantly expressed in cancers. However, the function and the underlying mechanisms of the NBAT-1 in colorectal carcinoma (CRC) remain unknown.

**Methods:**

Gene expression was detected by RT-qPCR. The influence of NBAT-1 on CRC was evaluated by the cell counting kit-8 (CCK-8) assay and an in vivo xenograft mouse model. The possible binding of NBAT-1 to miRNAs was predicted via the miRDB online tool and confirmed by a dual-luciferase reporter assay. Protein expression was detected by western blot.

**Results:**

NBAT-1 expression was significantly decreased in CRC tissues, especially in patients with oxaliplatin (OXA) resistance. NBAT-1 inhibited OXA-resistant CRC cell proliferation in vitro and tumor growth in vivo. The mechanism study revealed that NBAT-1 functioned as a competing endogenous RNA (ceRNA) of miR-4504. NBAT-1 bound miR-4504 and decreased miR-4504 expression in CRC cells. Furthermore, WW-and-C2-domain-containing protein family member 3 (WWC3) was identified as a target of miR-4504. Downregulation of NBAT-1 promoted miR-4504 expression and reduced the level of WWC3. Inhibition of WWC3 by NBAT-1 depletion inactivated Hippo signalling by inhibiting the phosphorylation of large tumor suppressor kinase 1 (LATS1) and yes-associated protein (YAP). Consistently, knockdown of NBAT-1 suppressed the expression of YAP transcriptional targets.

**Conclusions:**

These findings demonstrated that lncRNA NBAT-1 suppresses OXA-resistant CRC cell growth via inhibition of miR-4504 to regulate the WWC3/LATS1/YAP axis.

## 1. Introduction 

Colorectal cancer (CRC) is one of the most aggressive malignancies globally, with an increasing mortality rate [1–3]. Genetic or epigenetic mutations and chronic cirrhosis account for the majority of CRC cases [3]. Traditional antitumour therapies, including surgery and chemoradiotherapy, have significantly improved the clinical outcome of CRC patients. However, due to the resistance of chemotherapy, CRC is easy to recurrence, distant metastasis, and leads to poor survival [4]. Oxaliplatin (OXA) is commonly applied as a chemotherapy drug for the treatment of CRC patients, which reveals powerful efficiency to suppress the progression of CRC [5–8]. Nevertheless, the clinical application of OXA is seriously limited because of drug resistance. Therefore, exploring novel targets and developing alternative therapies to overcome the drug resistance of OX is one of the major challenges in the clinical CRC treatment.

lncRNAs are transcript regulators with more than 200 length nucleotides that epigenetically regulate gene expression, involving fundamental cellular physiological processes [9–11]. Notably, aberrant expression of lncRNAs is associated with CRC occurrence and progression [9, 11, 12]. lncRNAs exert a dual role as both tumour suppressors and oncogenes. Monitoring the alteration of lncRNA has shown certain diagnostic and prognostic significance in CRC progression [11, 12]. The most common mechanism of lncRNA in cancer regulation is acting as competing endogenous RNAs (ceRNAs) to sponge the function of microRNAs (miR or miRNA) through sharing their common response elements [13, 14]. miRNAs are characterized as small, single-stranded RNA transcripts without protein coding capacity [15, 16]. miRNAs induce target mRNA degradation or translation inhibition via binding the 3′-untranslated region (UTR) [17]. The ceRNA hypothesis between lncRNAs and miRNAs provides a broad control over gene expression and highlights the possibility for clarifying cancer progression at the transcriptional level. Neuroblastoma associated transcript-1 (NBAT-1) is a lncRNA. It was initially identified as a tumor suppressor in neuroblastoma [18]. Downregulated NBAT-1 promoted the malignancy of neuroblasts and was associated with the poorer prognosis of cancer patients [18]. Interestingly, the tumor suppressive roles of NBAT-1 have also been established in gastric cancer, lung cancer, clear cell renal cell carcinoma, and ovarian cancer [19–22]. These research studies highlight the potential therapeutic significance of NBAT-1 in cancer. However, the function of NBAT-1 in CRC, especially in the chemoresistance of CRC, has not been illustrated yet.

The Hippo pathway is an evolutionarily conserved signalling axis that plays important roles in organism development, cell proliferation, and epithelial-mesenchymal transition of cancer cells [23, 24]. The large tumor suppressor-1/2 (LATS1/2) kinase complex is the major component of the Hippo pathway, which phosphorylates the transcription coactivator yes-associated protein (YAP), sequesters YAP in the cytoplasm, and inhibits target gene transcription [25–27]. WW-and-C2-domain-containing protein 3 (WWC3), a homolog of the WWC gene family, was report to interact with LATS1, trigger the phosphorylation of LATS1, and suppress the Hippo pathway [28, 29]. Downregulation of WWC3 has been found in some cancers, thus WWC3 is recognized as a tumor suppressor [30–32]. Therefore, the involved mechanism by which WWC3 is regulated is critical for the interruption of cancer development.

In this study, NBAT-1 expression was found to be reduced in OXA-resistant CRC cells and tissues. Overexpression of NBAT-1 suppressed the malignant behaviours of CRC cells. A mechanism study revealed that NBAT-1 regulates the growth of OXA resistant-CRC cells by targeting WWC3 via suppressing miR-4504. These findings provided a novel molecular mechanism and an alternative treating strategy to overcome the chemoresistance of CRC.

## 2. Materials and Methods

### 2.1. CRC Tissues

50 cases of CRC patients who underwent surgery at the First Affiliated Hospital of Xi'an Jiaotong University between April 2012 and August 2014 were enrolled in this study. Among these 50 patients, 31 of them were OXA-sensitive, and the others (19 patients) have an OXA-resistant phenotype. The Ethics Committee of the First Affiliated Hospital of Xi'an Jiaotong University approved this study. Written informed consent was provided by all the participants.

### 2.2. Cell Culture

CRC cell lines HCT116 and SW480 and normal colorectal cells (CCD-112CoN) were purchased from ATCC (Manassas, VA, USA). OXA-resistant HCT116 and SW480 cells were obtained by continuously increasing exposure to OXA. Cells were cultured in DMEM (Gibco, EI Paso, Texas, USA) with 10% fetal bovine serum (FBS, Gibco). Cells were maintained at 37°C under a 5% (vol/vol) CO_2_ atmosphere.

### 2.3. CCK-8 Assay

OXA-resistant CRC cells (1,000 cells/well in 96 well plate) were exposed to different concentrations of OXA (Hengrui, Jiangsu, China) for 24 h. The proliferation ability of the CRC cells was evaluated using the Cell Counting Kit-8 (CCK-8; Beyotime) according to the manufacturer's guidelines. Briefly, 10 *μ*l of CCK-8 was added and incubated with the cells to be detected for 3 h at 37°C. The absorbance of each well at 450 nm was detected with BioTek's Synergy™ H4 and Synergy™ 2 multimode microplate readers (BioTek Instruments, Vermont, USA).

### 2.4. Cell Transfection

The scrambled small interfering siRNA-control and siRNA-NBAT-1, miR-scramble (negative control, miR-NC, 5′-UUCUCCGAACGUGUCACGUTT-3′), and miR-4504 mimics (5′-UGUGACAAUAGAGAUGAACAUG-3′) were purchased from GenePharma (Shanghai, China). When the cell confluence reached 60%, 50 nM oligonucleotides were transfected with Lipofectamine 2000 (Invitrogen, Carlsbad, CA, USA). Cells were lysed after 48 h of transfection for further analysis.

### 2.5. RT-qPCR

Total RNA was extracted with Trizol reagent (Quanxinquanyi, Shanghai, China). 0.5 *μ*g of the RNA was reversely transcribed into cDNA using PrimeScript™ RT Reagent Kit (Takara, Beijing, China). qPCR was performed with the SYBR-Green Real-time PCR Master Mix (TIANGEN, Beijing, China). The condition of the real-time PCR was set as follows: 96°C for 45 s, 42 cycles of 96°C for 10 s, and 60°C for 35 s. Expression of GAPDH or U6 mRNA was applied as an internal reference for normalization. The primers used in the studies were as follows: F-NBAT-1, 5′-ATTTCTGCTCCTGGGTCTTAC-3′ and R-NBAT-1, 5′-AGTGGCTTGTCTGTTAGAGTC-3′; F-GAPDH, 5′-AGGTCGGTGTGAACGGATTTG and R-GAPDH, 5′-GGGGTCGTTGATGGCAACA-3′; and F-WWC3, 5′-AGACAGTGCCAAGAGGTTGGAG-3′ and R–WWC3, 5′-CAGGCTCCTCGGCATCTTCGT-3′.

### 2.6. Western Blotting

20 *μ*g protein sample to be detected was loaded per well and separated by SDS-PAGE, transferred onto a membrane, and preblocked with 5% skimmed milk at room temperature (RT) for 1 h. Afterwards, the membrane was incubated with the corresponding primary antibody against-WWC3 (1 : 1000; ab243715, Abcam) or GAPDH (1 : 1000; sc-47724, Santa Cruz Biotechnology, USA), pLATS1 (Thr1079, #9159, Cell Signaling Technology, Shanghai, China), LATS1 (#9159, Cell Signaling Technology, Shanghai, China), pYAP (Ser127), YAP (#14074) overnight at 4°C, triplicate rinsed with TBS-T buffer (TIANGEN), and incubated with the corresponding horseradish peroxidase (HRP)-conjugated secondary antibody for 1h. After triplicate washing with TBS-W buffer, the blot protein was visualized with an enhanced chemiluminescence kit (Thermo Fisher, Waltham, MA, USA).

### 2.7. Duel-Luciferase Reporting Assay

NBAT-1 and miR-4504 potential targets were predicted with the miRDB MicroRNA Target Prediction Database (http://mirdb.org/), respectively. For the dual-luciferase reporter assay, NBAT-1 fragments or the 3′-UTR of WWC3 that carried miR-4504 binding were inserted into the pMIR-reporter vector (Promega, Madison, Wisconsin, USA). OXA-resistant CRC cells were cotransfected with pMIR-wild-type (WT)/mutant (Mut) vector (100 ng) with miR-4504 mimics or miR-NC (50 nM) using the Lipofectamine 2000. After transfection for 48 h, Renilla and Firefly luciferase activity was detected using the Dual-Luciferase Reporter Assay System (Promega).

### 2.8. Cell Apoptosis

CRC cell apoptosis was detected using the propidium iodide (PI) and FITC/Annexin V Apoptosis kit (BD Biosciences, San Jose, CA, USA). After transfection for 48 h, cells were harvested and resuspended in 400 *μ*l of binding buffer (from the kit). Cells were incubated with 5 *μ*l of Annexin V-FITC for 15 min at room temperature, followed by PI staining for 10 min in the dark. The apoptotic profile of the cells was detected by FACSCalibur™ Flow Cytometer (BD Biosciences).

### 2.9. In Vivo Xenograft Mice Assay

BALB/c nude mice (5–6 weeks, female) were obtained from the Charles River (Beijing, China) and housed under a 12 h of light/dark cycle with free access to water and food. CRC cells (3 × 10^6^) with stably expressed NBAT-1 or control vector were subcutaneously injected. Tumor growth was monitored with a caliper every 3 days. Mice were sacrificed via cervical dislocation and the tumor formation was carefully removed.

### 2.10. Statistical Analysis

The experimental data were presented as the mean ± standard deviations (SD) and analyzed using the GraphPad Prism. Student's *t*-test or one-way analysis of variance (ANOVA) followed by Tukey's test was run to determine the significance (*P* < 0.05).

## 3. Results

### 3.1. NBAT-1 Was Downregulated in OXA-Resistant CRC Tissues and Cells

To investigate the potential involvement of NBAT-1 in CRC, NBAT-1 expression in CRC tissues and paired adjacent normal tissues was determined. As indicated in Figure 1(a), NBAT-1 level was significantly lower in CRC tissues than that of the noncancerous tissues. Downregulated NBAT-1 expression was also observed in the CRC cell lines HCT116 and SW480 (Figure 1(b)). These results suggested the downregulation of NBAT-1 in CRC. Furthermore, to discover whether dysregulation of NBAT-1 was associated with the OXA-resistance of CRC, the abundance of NBAT-1 in OXA-resistant and OXA-sensitive CRC tissues was compared. RT-qPCR analysis showed that NBAT-1 was markedly lower in OXA-resistant CRC samples than in OXA-sensitive tissues (Figure 1(c)). Moreover, NBAT-1 was also lowerly expressed in OXA-resistant HCT116 and SW480 cell lines compared with their parental cells (Figure 1(d)). These results indicated the downregulation of NBAT-1 in CRC OXA-resistance.

### 3.2. NBAT-1 Overexpression Inhibited OXA-Resistant CRC Cell Growth

Before evaluating the effects of NBAT-1 on chemoresistance of CRC, the proliferation of OXA-sensitive (normal) HCT116 and SW480, as well as OXA-resistant HCT116 (HCT116/OXA) and SW480 (SW480/OXA) cells were compared. The CCK-8 assay showed that the cellular viability of HCT116/OXA and SW480/OXA was significantly higher compared with their parental HCT116 and SW480 cells at a 6 *μ*M dose of OXA level (Figure 2(a)). The NBAT-1-expression plasmid was transfected into both HCT116/OXA and SW480/OXA cells to upregulate NBAT-1. The overexpression of NBAT-1 was validated by RT-qPCR (Figure 2(b)). Interestingly, overexpressed NBAT-1 significantly suppressed either the HCT116/OXA or the SW480/OXA cell proliferation (Figures 2(c) and 2(d)). To investigate the influence of the cell cycle on the enhanced OXA-resistant, we performed FACS analysis in the NBAT-1-overexpressed HCT116/OXA and SW480/OXA cells. Notably, NBAT-1 overexpression significantly inhibited the cell cycle of the OXA-resistant CRC cells with increased accumulation in the G_1_ phase (Figures 2(e) and 2(f)). These results demonstrated that NBAT-1 suppressed OXA-resistant CRC cell growth.

To provide more evidence to support the antioncogenic activity of NBAT-1 in the OXA-resistance of CRC, a xenograft mouse model was established by subcutaneously injecting either the HCT116/OXA or the SW480/OXA cells transfected with the NBAT-1 expressing vector. The NBAT-1 overexpression in the xenograft tumors was validated by RT-qPCR in the CRC xenograft mice models (Figure 2(g)). Consistently, NBAT-1 overexpression significantly reduced the tumor volume in both the HCT116/OXA and the SW480/OXA xenograft mouse models (Figure 2(h)). Overall, these results demonstrated that NBAT-1 suppressed the tumor growth of either the OXA-resistant CRC cells or the CRC mice models, indicating the antioncogenic activity of NBAT-1 in OXA-resistant CRC.

### 3.3. NBAT-1 Negatively Regulated miR-4504 in CRC

Based on the ceRNA hypothesis, the possible binding miRNAs to the BNTA-1 were predicted using the miRDB MicroRNA Target Prediction Database (http://mirdb.org/). miR-4504 was found to interact with NBAT-1 (Figure 3(a)). Further investigation indicated that the expression of miR-4504 was significantly increased in the OXA-resistant CRC tissues compared with that of OXA-sensitive CRC tissues (Figure 3(b)). Similarly, a higher level of miR-4504 was also found in the OXA-resistant CRC cells than their parental cells (Figure 3(c)). To confirm the binding between miR-4504 and NBAT-1, a dual-luciferase reporter assay was performed with HCT116/OXA and SW480/OXA cells cotransfected with wild-type (WT) or mutant NBAT-1 and miR-4504 mimics. Clearly, overexpression of miR-4504 markedly reduced the luciferase activity of WT but not in the mutant NBAT-1 (Figures 3(d) and 3(e)). RT-qPCR assay was performed to determine the level of miR-4504 with the transfection of NBAT-1. The data indicated that miR-4504 expression was significantly reduced after overexpression of NBAT-1 in HCT116/OXA and SW480/OXA (Figure 3(f)). These results suggested that NBAT-1 was bound with miR-4504 and inhibited the expression of miR-4504 in the OXA-resistant CRC cells.

To evaluate whether the antioncogenic activity of NBAT-1 was mediated by miR-4504 inhibition in the chemoresistance of CRC, HCT116/OXA, and SW480/OXA cells were cotransfected with NBAT-1 and miR-4504 mimics, and then the cell proliferation was determined. As shown in Figures 3(g) and 3(h), overexpression of NBAT-1 obviously reduced cellular proliferation of the OXA-resistance of CRC cells. While transfection of miR-4504 significantly abrogated the proproliferative effects of NBAT-1 in both the HCT116/OXA and the SW480/OXA cells.

### 3.4. WWC3 Was a Target Factor of miR-4504 in CRC

To understand the molecular mechanisms by which miR-4504 mediates the antioncogenic activity of NBAT-1 in the CRC chemoresistance, the potential targets of the miR-4504 were predicted using the miRDB database. The data showed that miR-4504 contained complementary binding sites within the 3′-UTR of WWC3 (Figure 4(a)). To confirm this finding, HCT116/OXA and SW480/OXA cells were cotransfected with the dual-luciferase reporter vector harboring with either the WT or Mut 3′-UTR of WWC3 and miR-4504 mimics. Notably, overexpression of miR-4504 significantly reduced the luciferase activity of the cells expressing WT WWC3 (Figures 4(b) and 4(c)), suggesting the specific interaction between the miR-4504 and the 3′-UTR of WWC3. To further determine the effects of miR-4504 on WWC3, the expression level of WWC3 was detected by RT-qPCR and western blot, respectively, in the HCT116/OXA and SW480/OXA cells. Both the mRNA and protein abundance of the WWC3 was significantly reduced by the overexpression of miR-4504 (Figures 4(d) and 4(e)). These findings revealed that WWC3 was a target of miR-4504 in CRC.

To investigate the correlation between WWC3 with the OXA-resistance of CRC, the level of WWC3 in OXA-resistant or sensitive CRC tissues was compared. As indicated in Figure 4(f), WWC3 expression was markedly lower in the OXA-resistant CRC tissues than in OXA-sensitive tissues. Additionally, since NBAT-1 suppressed miR-4504, we also checked the effect of NBAT-1 on the expression of WWC3. Interestingly, the mRNA level of WWC3 was decreased after silencing of NBAT-1 in either the HCT116/OXA or the SW480/OXA cells (Figure 4(g)). Consistently, the protein expression of WWC3 was also reduced with the NBAT-1 knockdown (Figure 4(h)). Overall, these data indicated that NBAT-1 regulated the expression of WWC3 via sequestering miR-4504 in OXA-resistant CRC cells.

### 3.5. NBAT-1 Depletion Activated the Hippo Pathway

Previous studies demonstrated WWC3 as an upstream activator of the Hippo pathway by interacting with LATS1 and promoting the phosphorylation of YAP1 [33]. Given the relationship between WWC3 and NBAT-1, the effects of NBAT-1 on Hippo signalling were evaluated by detection of the phosphorylation of LATS1. The results showed that NBAT-1 depletion by si-BAT-1 reduced the phosphorylation of LATS1 in both HCT116/OXA and SW480/OXA cells (Figure 5(a)). Consistent with the inaction of LAST1, the phosphorylation of YAP was also decreased with the knockdown of NBAT-1 (Figure 5(a)). It has been reported that once phosphorylated, YAP was sequestered in the cytoplasm and inactivated the transcriptional activity of YAP. As shown in Figures 5(b) and 5(c), NBAT-1 knockdown significantly increased the expression of connective tissue growth factor (CTGF), AXL, and cysteine-rich61 (CYR61), which are the established transcriptional targets of YAP [34]. Collectively, these results identified NBAT-1 as a novel regulatory of the Hippo pathway.

## 4. Discussion

CRC is one of the most prevalent cancers and a leading cause of cancer-related death [11]. Currently, surgical section combined with chemotherapy is the main option for the treatment of CRC [4]. However, there were still a lot of patients responding poorly to the chemotherapy, which results into the tumor relapse with a more aggressive and chemoresistant phenotype. Therefore, understanding the underlying molecular mechanisms that contribute to the chemoresistance of CRC is important to overcome the obstacles of chemotherapy and improve the prognosis of CRC patients. Here, we found that NBAT-1 has an antioncogenic activity in OXA-resistant CRC tissues and cells, indicating the potential significance of NBAT-1 in the development and chemoresistance of CRC.

Exploring the roles of lncRNAs in CRC has attracted much attention and is becoming a hot spot to understand the molecular mechanisms that may be responsible for the progression of cancer [11]. NBAT-1 was initially identified as a lncRNA that was downregulated in neuroblastoma and predicted a poor clinical outcome of patients [18]. Loss of NBAT-1 contributed to the aggressive progression of neuroblastoma via promoting the proliferation and impairing the differentiation of neuronal precursors. Recently, the reduced expression and antioncogenic activity of NBAT-1 have also been uncovered by increasing studies [35–38]. The decreased level of NBAT-1 was associated with the poor prognosis of clear cell renal cell carcinoma (ccRCC) patients, exhibiting the clinical significance of NBAT-1 in the diagnosis and treatment of ccRCC [19]. Additionally, lower expression of NBAT-1 was also found in gastric cancer and lung cancer, where overexpression of NBAT-1 suppressed the oncogene and predicted a favourable prognosis of cancer patients [20, 21]. In this study, NBAT-1 was downregulated in OXA-resistant CRC tissues. Overexpression of NBAT-1 suppressed the proliferation and cell cycle progression of OXA-resistant CRC cells. Notably, in vivo data also demonstrated that highly expressed NBAT-1 inhibited the growth of chemoresistant CRC cells. These findings indicated the antioncogenic activity of NBAT-1 in the chemoresistance of CRC.

miRNA is closely associated with the occurrence and progression of cancers via acting as an oncogene or tumor suppressor. Based on the ceRNA mechanism, lncRNA sponges miRNA and antagonizes the inhibiting effect of miRNA against the target genes [13]. In this study, miR-4504 was predicted and confirmed as a binding target of NBAT-1. miR-4504 was overexpressed in OXA-resistant CRC tissues. This pro-oncongenic activity of miR-4504 has not been revealed before in the development and chemoresistance of CRC. Decreased expression of WWC3 was found in lung cancer and associated with the poor survival of cancer patients [29, 31]. In this study, NBAT-1 silencing reduced the level of WWC3 in the OXA-resistant CRC cells. Lower expression of WWC3 by NBAT-1 depletion decreased the phosphorylation of LATS1 and YAP, thus inhibiting the Hippo pathway. These findings demonstrated that NBAT-1 regulated WWC3 via sequestering miR-4504, and consequently, modulated the phenotype of OXA-resistant CRC cells.

Although most studies on BNAT-1 and cancer are still in early stages, our data showed that lower NBAT-1 is favorable for CRC growth. Therefore, NBAT-1 or miR-4504 detection could be applied clinically to evaluate the CRC growth state and prognosis during the treatment of CRC. Indeed, Yuan Gao and Jianping Chen have investigated the regulation of lncRNA NBAT-1 on gastric cancer (GC) development and prognosis [22]. They found that decreased lncRNA NBAT-1 is associated with poor prognosis.

In summary, our study showed the reduced expression of NBAT-1 in OXA-resistant CRC tissues and cells. Overexpressed NBAT-1 suppressed the malignant phenotypes of OXA-resistant CRC cells via suppressing miR-4504 to upregulate WWC3 and inhibit the oncogenic Hippo signalling pathway. This study demonstrated the novel antioncogenic mechanism of NBAT-1 in the chemoresistance of CRC, providing a novel target point for the therapy of CRC.

## Figures and Tables

**Figure 1:** NBAT-1 was reduced in OXA-resistant CRC. (a) NBAT-1 mRNA expression in CRC tissues and paired noncancerous tissues was compared by RT-qPCR. (b) NBAT-1 levels in normal colorectal cells (CCD-112CoN) and CRC cell lines (HCT116 and SW480) were examined via RT-PCR analysis. NBAT-1 mRNA expression in OXA-resistant CRC tissues (c) and cells (d) were detected by qRT-PCR. OXA-sensitive CRC tissues and parent cells (HCT116 and SW480) were used as controls. ^*∗∗∗*^*P* < 0.001. Each data of B and D came from three independent assays.

**Figure 2:** NBAT-1 inhibited the OXA-resistant CRC growth. (a) OXA-resistant CRC and parental CRC cells were treated with indicated increasing doses of OXA for 48 h and the cell survival was determined by the CCK8 assay. (b) Expression levels of NBAT-1 were detected by RT-qPCR in the HCT116/OXA and SW480/OXA cells transfected with either empty vector or NBAT-1 expressing vector. (C, D) Cellular proliferation of NBAT-1-transfected HCT116/OXA (c) and SW480/OXA (d) cells was analyzed by the CCK-8 assay. (E, F) Cell cycle was analyzed by FACS flow cytometry in the NBAT-1-transfected and empty vector-transfected HCT116/OXA (e) and SW480/OXA (f) cells. (g) HCT116/OXA and SW480/OXA cells transfected with control lentivirus vector or NBAT-1 lentivirus were implanted into the flanks of nude mice. The NBAT-1 mRNA expression was detected by RT-qPCR in the grown xenograft tumors. (h) Tumor volume were measured at indicated days in the HCT116/OXA and SW480/OXA transfected with NBAT-1 or control xenograft mice. ^*∗∗*^*P* < 0.01, ^*∗∗∗*^*P* < 0.001. Each data came from three independent assays.

**Figure 3:** NBAT-1 suppressed miR-4504 in OXA-resistant CRC cells. (a) The predicted binding sequence of NBAT-1 with miR-4504 in miRDB MicroRNA Target Prediction Database (http://mirdb.org/). (b) miR-4504 expression was detected by qRT-PCR in the OXA-resistant and sensitive CRC tissues. (c) miR-4504 expression was detected by qRT-PCR in the OXA-resistant CRC cells. (D, E) Interaction between the miR-4504 and NBAT-1 was analyzed by dual-luciferase reporter assay in the HCT116/OXA (d) or SW480/OXA (e) cells cotransfected with wild-type (WT) or mutant of NBAT-1 and miR-4504 mimics. miR-scramble (miR-NC) was used as negative controls. (f) miR-4504 expression was detected by qRT-PCR in the HCT116/OXA and SW480/OXA OXA-resistant CRC cells transfected with NBAT-1 or empty vector. (G, H) Cellular proliferation was assayed by CCK8 assay in the HCT116/OXA (g) and SW480/OXA (h) cells. ^*∗∗*^*P* < 0.01, ^*∗∗∗*^*P* < 0.001. Each data came from three independent assays.

**Figure 4:** miR-4504 targeted and inhibited WWC3 in OXA-resistant CRC cells. (a) Binding sites of WWC3 3′-UTR with miR-4504. (B, C) Luciferase activity of the HCT116/OXA (b) and SW480/OXA (c) cells transfected with miR-4504 or miR-NC and WWC3 or mutated WWC3 were detected in a dual-luciferase assay system. (D, E) WWC3 protein (d) and mRNA (e) levels were detected by Western blot and qRT-PCR in the miR-4504 overexpressed HCT116/OXA and SW480/OXA cells. (f) WWC3 mRNA expression was analyzed by qRT-PCR in the OXA-resistant CRC tissues and the OXA-sensitive tissues. (G, H) WWC3 mRNA (g) and protein (h) expression were evaluated by qRT-PCR (G) and western blot (H) in the si-NBAT-1-transfected HCT116/OXA and SW480/OXA cells. ^*∗∗∗*^*P* < 0.001. Each data came from at least three independent assays.

**Figure 5:** Inhibition of NBAT-1 suppressed Hippo signalling. (A) Phosphorylation of LATS1 and YAP was analyzed by western blot in the siRNA-NBAT-1-transfected HCT116/OXA and SW480/OXA cells. (B, C) ALX, CYR61, and CTGF proteins expression were assayed by western blot. ^*∗∗∗*^*P* < 0.001. Each data came from at least three independent assays.

## Data Availability

The data used to support the findings of this study are available from the corresponding author upon request.
